# Increased Risk of Benign Prostate Hyperplasia (BPH) in Patients with Gout: A Longitudinal Follow-Up Study Using a National Health Screening Cohort

**DOI:** 10.3390/diagnostics14010055

**Published:** 2023-12-26

**Authors:** Woo Jin Bang, Hyo Geun Choi, Ho Suk Kang, Mi Jung Kwon, Ji Hee Kim, Joo-Hee Kim, So Young Kim

**Affiliations:** 1 Department of Urology, Hallym University Sacred Heart Hospital, Hallym University College of Medicine, Anyang 14068, Republic of Korea; yybbang@hallym.or.kr; 2 Suseoseoulent Clinic, Seoul 06349, Republic of Korea; pupen@naver.com; 3 Division of Gastroenterology, Department of Internal Medicine, Hallym University Sacred Heart Hospital, Anyang 14068, Republic of Korea; putamenn@hanmail.net; 4 Department of Pathology, Hallym University Sacred Heart Hospital, Hallym University College of Medicine, Anyang 14068, Republic of Korea; mulank99@hallym.or.kr; 5 Department of Neurosurgery, Hallym University Sacred Heart Hospital, Hallym University College of Medicine, Anyang 14068, Republic of Korea; kimjihee@hallym.or.kr; 6 Department of Medicine, Hallym University Sacred Heart Hospital, Hallym University College of Medicine, Anyang 14068, Republic of Korea; luxjhee@hallym.or.kr; 7 Department of Otorhinolaryngology-Head & Neck Surgery, CHA Bundang Medical Center, CHA University, Seongnam 13488, Republic of Korea

**Keywords:** benign prostate hyperplasia, gout, risk factors, cohort studies, epidemiology

## Abstract

A previous study reported a high risk of benign prostatic hyperplasia (BPH) in patients with gout. This study intended to evaluate the risk of BPH in gout patients. A total of 514,866 Korean National Health Insurance Service—Health Screening Cohorts were retrieved from 2002 to 2019. Among these individuals, 14,961 gout patients and 58,764 control participants were matched based on demographic factors. The incidence of BPH during the follow-up periods was collected for both the gout and control groups. The risk of BPH was analyzed using stratified Cox proportional hazard models, and hazard ratios (HRs) and 95% confidence intervals (CIs) were calculated. Secondary analyses were conducted based on demographic factors and comorbidities. The incidence of BPH was 23.40% in gout patients and 20.70% in control participants. In the adjusted model, the HR of BPH was 1.13-fold higher in gout patients than in the control group (95% CI = 1.09–1.18). Compared with the ≥60-year-old group, the <60-year-old group demonstrated a higher HR for BPH in gout patients (1.19 [1.13–1.24] vs. 1.07 [1.01–1.13]). The risk of BPH in gout patients was consistent according to various comorbidities. Patients with gout demonstrated a greater risk of BPH than participants without gout. The young adult population had a higher risk of BPH related to gout.

## 1. Introduction

Benign prostatic hyperplasia (BPH) is histologically defined as the abnormal proliferation of epithelial and stromal cells in the prostate gland, which encompasses the proximal urethra [1]. Approximately 26.2% of the population is estimated to suffer from BPH [2]. The prevalence of BPH increases with age, as more than 50% of the population older than 60 years has BPH [3]. In Korea, approximately 20.0% of males are diagnosed with BPH, and the prevalence of BPH is as high as 26.6% in populations older than 70 years [4]. To relieve the difficulties in emptying and retaining patients, several types of medical and surgical approaches are employed [5,6,7]. Because many of these treatments cannot reverse the changes in prostate hyperplasia, preventive management and the delineation of the risk factors of BPH are important. A number of lifestyle factors, such as obesity; high intake of carbohydrates, fat, protein, and sugar; smoking; alcohol consumption; and sedentary behavior, have been suggested to increase the risk of BPH [8]. In addition, comorbidities, including metabolic disorders such as diabetes and related medications, hypertension, and dyslipidemia, are purportedly associated with increased susceptibility to BPH [9].

Gout is one of the most common inflammatory arthritis types. Uric acid deposits mainly originate from chronic hyperuricemia, which causes inflammatory arthritis [10]. In the U.S., the prevalence of gout is approximately 5.9% in men and 2.0% in women [3]. In Korea, the incidence of gout was estimated to be approximately 1.94 (95% confidence intervals (CI) = 1.93–1.95) per 1000 persons, and the incidence of gout was calculated to be approximately 7.58 (7.55–7.60) [11]. Because gout also involves the perturbation of metabolism, which results in the deposition of urate crystals and inflammation, patients with gout may be more vulnerable to the development of BPH. Indeed, a previous cohort study reported a 1.3 times greater risk of BPH in patients with gout [12]. In particular, a young male population aged >60 years demonstrated a high risk of BPH among gout patients but not in a population older than 60 years. Moreover, an association between uric acid levels and the risk of BPH has been suggested. A population cohort study reported a lower risk of BPH related to urate-lowering medication, such as allopurinol [13]. Allopurinol use lowers the risk of BPH in terms of medication, diagnosis, and surgery (HR = 0.81 [0.75–0.88], 0.78 [0.71–0.86], and 0.67 [0.58–0.76]) [13].

The present study hypothesized that patients with gout, including those in the older age group, have a greater risk of BPH in the adult population. Moreover, we investigated the risk of BPH in gout patients according to comorbid conditions and lifestyle factors. This study used large, nationwide population data in Korea, which reduced selection bias due to the limited number of study populations.

## 2. Materials and Methods

### 2.1. Exposure (Gout)

Gout was defined as occurring in participants who visited the clinic or hospital with a diagnosis of gout (International Classification of Diseases (ICD-10): M10) ≥ 2 times. These methods were modified from the previous study.

### 2.2. Outcome (Definition of Benign Prostatic Hyperplasia)

Benign prostatic hyperplasia (BPH) was defined using International Classification of Diseases 10 code (ICD-10 code) N40 from 2002 through 2019. Among them, we selected the participants who were treated ≥2 times and participants who were diagnosed with BPH with an exam (claim codes: C4280, E7050, EY521, EY522, EB451) following our previous studies.

### 2.3. Participant Selection

A detailed description of the Korean National Health Insurance Service—Health Screening Cohort data was provided recently in [14].

Gout participants were selected from 514,866 participants with 895,300,177 medical claim codes from 2002 to 2019 (*n* = 27,313). The control group included participants who were not diagnosed with gout between 2002 and 2019 (*n* = 487,553). To select gout participants who were diagnosed for the first time, gout participants diagnosed in 2002 were excluded (washout periods, *n* = 2470). To select only men, females were excluded (*n* = 5281). Control participants were also excluded if they were diagnosed with M10 per the International Classification of Diseases 10 (ICD-10) code once or if they were females (*n* = 212,229). In both the gout and control groups, participants who had a history of BPH before the index date were excluded. In the gout group, 4870 participants were excluded. Participants who did not have a blood pressure record were excluded (*n* = 1). Gout participants were 1:4 matched with control participants for age, sex, income, and region of residence. To prevent selection bias when selecting the matched participants, the control participants were sorted using a random number order and were subsequently selected from top to bottom. It was assumed that the matched control participants were evaluated at the same time as each matched gout participant (index date). Therefore, participants in the control group who died before the index date were excluded. During the matching procedure, 216,560 control participants were excluded. Finally, 14,691 gout participants were 1:4 matched with 58,764 control participants (Figure 1).

### 2.4. Covariates

Age was divided into 5-year intervals: 40–44… and 85+ years. A total of 10 age groups were specified. Income groups were classified into 5 classes (class 1 (lowest income) to class 5 (highest income)). The regions of residence were grouped into urban (Seoul, Busan, Daegu, Incheon, Gwangju, Daejeon, and Ulsan) and rural (Gyeonggi, Gangwon, Chungcheongbuk, Chungcheongnam, Jeollabuk, Jeollanam, Gyeongsangbuk, Gyeongsangnam, and Jeju) areas.

Tobacco smoking was categorized based on the participant’s current smoking status (nonsmoker, past smoker, and current smoker). Alcohol consumption was categorized on the basis of the frequency of alcohol consumption (<1 time a week and ≥1 time a week). Obesity was measured using BMI (body mass index, kg/m^2000^). BMI was categorized as <18.5 (underweight), ≥18.5 to <23 (normal), ≥23 to <25 (overweight), ≥25 to <30 (obese I), and ≥30 (obese II) based on the Asia–Pacific criteria following the Western Pacific Regional Office (WPRO) [15]. Systolic blood pressure (mmHg), diastolic blood pressure (mmHg), fasting blood glucose (mg/dL), and total cholesterol (mg/dL) were measured.

The Charlson Comorbidity Index (CCI) was used to measure disease burden using 17 comorbidities. A score was given to each participant depending on the severity and number of diseases. The CCI was measured as a continuous variable (0 (no comorbidities) to 29 (multiple comorbidities)) [16].

### 2.5. Statistical Analyses

The standardized difference was used to compare the percentages of patients with different general characteristics between the gout and control groups.

Stratified Cox proportional hazard models were used to assess the hazard ratios (HRs) and 95% confidence intervals (CIs) of gout for BPH. Crude (simple) and adjusted (obesity, smoking, alcohol consumption, systolic blood pressure, diastolic blood pressure, fasting blood glucose, total cholesterol, and CCI scores) models were used in these analyses, and the 95% CI was calculated. In these analyses, age, sex, income, and region of residence were stratified. K—M curves and logrank tests were used.

For the subgroup analyses using the stratified Cox-proportional hazards model, we divided participants by age, sex, obesity, and fasting blood glucose.

We performed additional subgroup analyses using the unstratified Cox-proportional hazards model. We divided participants by income, region of residence, smoking status, alcohol consumption, systolic blood pressure, diastolic blood pressure, total cholesterol, and CCI scores.

Two-tailed analyses were performed, and *p*-values less than 0.05 were considered to indicate statistical significance. SAS version 9.4 (SAS Institute, Inc., Cary, NC, USA) was used for the statistical analyses.

## 3. Results

A total of 23.40% (3438/14,691) of the gout patients and 20.70% (12,163/58,764) of the control participants were diagnosed with BPH (sd = 0.07; Table 1). The distributions of obesity groups, smoking status, alcohol consumption, systolic blood pressure, diastolic blood pressure, fasting blood glucose, total cholesterol, and CCI score were different between the BPH and control groups.

The gout patients demonstrated a 1.15 times greater risk of BPH than did the control individuals in the crude analysis (95% CI = 1.11–1.20, *p* < 0.001; Table 2). After adjusting for covariables, the risk of BPH was 1.13 times greater in the gout patients than in the control individuals (95% CI = 1.09–1.18, *p* < 0.001; Figure 2).

According to age, the younger age group (<60 years old) showed a higher risk of BPH than the older age group (≥60 years old) for gout patients (HR = 1.19, 95% CI = 1.13–1.25 for <60-year-old group and HR = 1.07, 95% CI = 1.01–1.13 for ≥60-year-old group). The male, low or high income, urban or rural residence, normal weight, overweight, obese, nonsmoker, past and current smoker, and alcohol consumption <1 times a week or ≥1 times a week subgroups and CCI scores of zero or one indicated a higher risk of BPH in gout patients.

## 4. Discussion

The risk of BPH was greater in patients with gout in the present study. Although the risk of BPH was greater in the young adult population, the old population also demonstrated an elevated risk for BPH in gout patients in the present study.

Chronic hyperuricemia in gout patients can increase the subsequent risk of BPH. It has been suggested that oxidative stress can induce BPH by activating the inflammasome in response to uric acid [17]. The impact of high levels of uric acid in serum on the proliferation of prostate cancer cells was suggested to be mediated by urate transporters in [18]. In addition, there is supporting evidence that reducing serum urate levels decreases the risk of BPH [13]. A cohort study revealed that high serum uric acid levels are associated with a low risk of lower urinary tract symptoms [19]. Thus, it can be presumed that there is a close relationship between uric acid levels and BPH. Most patients with gout are exposed to chronic hyperuricemia, which induces the accumulation of urate crystals in articular and nonarticular areas [20]. In addition to the deposition of urate in articular areas, high levels of serum urate can result in the modulation of prostate cells and may increase the risk of BPH.

In addition to hyperuricemia, systemic inflammatory conditions and abnormalities in testosterone levels can mediate the elevated risk of BPH in gout patients. Both gout and BPH are accompanied by systemic inflammation. The activation of the NOD-, LRR-, and pyrin domain-containing protein 3 (NLRP3) inflammasome, which initiates inflammatory cascades involving interleukin-1β and other inflammatory cytokines, is known for acute gout attacks [21]. In addition to the NLRP3-related pathway, more than 200 genes have been suggested to be dysregulated in gout patients; these genes are mainly associated with inflammation, cytokines, and chemokine activation [22]. The pathophysiology of BPH also includes inflammation and metabolic derangements [23,24]. Thus, metabolic and inflammatory dysfunctions in gout patients can increase vulnerability to BPH. Moreover, testosterone may mediate the link between gout and BPH. A low level of testosterone was suggested to be related to BPH [10]. Low testosterone levels have also been reported to be associated with hyperuricemia in males [25]. Thus, abnormal testosterone levels may link hyperuricemia in gout patients with the risk of BPH.

Decreased physical activity due to arthritis and acute symptoms in gout patients could increase the risk of BPH. A follow-up study demonstrated an increased risk of BPH in participants with low physical activity [26]. Physical activity was negatively associated with BPH incidence (OR = 0.75, 95% CO = 0.67 = 0.85) [26]. Thus, a sedentary lifestyle due to arthritic symptoms in gout patients can impose an increased risk of BPH in these populations.

The old population demonstrated a lower risk of BPH related to gout than the younger population in the present study. This may be explained by the multiple contributing factors to the development of BPH in the older population. For instance, a certain pathology in the aging process, mitochondrial dysfunction, may contribute to fibrosis and dysfunction in the prostate, which results in BPH [27]. According to our subgroup analyses, the presence or absence of comorbidities and lifestyle factors did not modify the association between gout and BPH. Therefore, we can assume that the risk of BPH associated with gout may be solid and multifactorial and cannot be ruled out given these comorbidities and lifestyle factors.

This study analyzed a large, nationwide cohort population. A sufficient number of control participants can be fooled without potential selection bias. Because all Koreans are legally registered with the national health insurance system and their medical records must be recorded and monitored by the government, the reliability of this study can be guaranteed.

However, there are several limitations concerning potential bias and uncertainty in the present study. Because the data were collected from clinics, hidden patients who did not visit clinics were missed in the present study. In addition, the types and severity of gout were heterogeneous in the present study. A previous study reported that gouty nephropathy patients, other than those with other types of gout, including gouty arthropathy and gouty tophi, demonstrated a high risk of BPH [12]. Thus, the differentiation of gout types can specify the relationship between gout and BPH in future studies. The severity and treatment history of BPH also varied among the study populations. Several surgical modalities and other modalities, including uroflowmetry, are used to treat BPH according to the established guidelines [6,7,28]. In Korea, medication has been reported to be the most prevalent therapy for BPH patients (98.77%) [29]. A previous study reported that medication for BPH was associated with the incidence of gout [30,31]. Therefore, medication history can influence the relationship between gout and BPH in this study. Although this study analyzed numerous variables and secondary analyses were conducted, confounders may remain in the current study. Because this study was based on a Korean population, ethnic or regional differences may be possible regarding the association between the two diseases. Further studies are warranted to explore the different types of gout and their associations with BPH considering the effects of medication on this relationship and investigating ethnic or regional variations in this association.

## 5. Conclusions

Patients with gout had a higher risk of BPH in the adult population. The elevated risk of BPH in gout patients was independent of lifestyle factors and comorbid conditions. Clinicians may need to consider the potentially increased risk of BPH when managing patients with gout and the need for early monitoring or intervention.

## Figures and Tables

**Figure 1:** A schematic illustration of the participant selection process used in the present study. Among a total of 514,866 participants, 14,691 gout participants were matched with 58,764 control participants for age, sex, income, and region of residence.

**Figure 2:** The risk of benign prostate hyperplasia in patients with gout compared with the control group.

**Table 1:** Patient general characteristics.

Characteristics	Total Participants		
	Gout	Control	Standardized Difference
Age (years old) (*n*, %)			0.00
40–44	497 (3.38)	1988 (3.38)	
45–49	1660 (11.30)	6640 (11.30)	
50–54	2654 (18.07)	10,616 (18.07)	
55–59	3136 (21.35)	12,544 (21.35)	
60–64	2440 (16.61)	9760 (16.61)	
65–69	1910 (13.00)	7640 (13.00)	
70–74	1288 (8.77)	5152 (8.77)	
75–79	752 (5.12)	3008 (5.12)	
80–84	280 (1.91)	1120 (1.91)	
85+	74 (0.50)	296 (0.50)	
Sex (*n*, %)			0.00
Male	14,691 (100.0)	58,764 (100.0)	
Income (*n*, %)			0.00
1 (lowest)	1901 (12.94)	7604 (12.94)	
2	1807 (12.30)	7228 (12.30)	
3	2245 (15.28)	8980 (15.28)	
4	3127 (21.29)	12,508 (21.29)	
5 (highest)	5611 (38.19)	22,444 (38.19)	
Region of residence (*n*, %)			0.00
Urban	6268 (42.67)	25,072 (42.67)	
Rural	8423 (57.33)	33,692 (57.33)	
Obesity † (*n*, %)			0.33
Underweight	173 (1.18)	1508 (2.57)	
Normal	3395 (23.11)	20,146 (34.28)	
Overweight	4067 (27.68)	16,689 (28.40)	
Obese I	6442 (43.85)	19,123 (32.54)	
Obese II	614 (4.18)	1298 (2.21)	
Smoking status (*n*, %)			0.03
Nonsmoker	6226 (42.38)	24,436 (41.58)	
Past smoker	2460 (16.74)	9126 (15.53)	
Current smoker	6005 (40.88)	25,202 (42.89)	
Alcohol consumption (*n*, %)			0.14
<1 time a week	6931 (47.18)	31,880 (54.25)	
≥1 time a week	7760 (52.82)	26,884 (45.75)	
Systolic blood pressure (*n*, %)			0.20
<120 mmHg	3779 (24.22)	14,711 (25.43)	
120–139 mmHg	7850 (50.32)	29,617 (51.19)	
≥140 mmHg	3972 (25.46)	13,526 (23.38)	
Diastolic blood pressure (*n*, %)			0.19
<80 mmHg	5905 (37.85)	23,356 (40.37)	
80–89 mmHg	5985 (38.36)	22,464 (38.83)	
≥90 mmHg	3711 (23.79)	12,034 (20.80)	
Fasting blood glucose (*n*, %)			0.03
<100 mg/dL	9336 (59.84)	31,992 (55.30)	
100–125 mg/dL	4680 (30.00)	18,955 (32.76)	
≥126 mg/dL	1585 (10.16)	6907 (11.94)	
Total cholesterol (*n*, %)			0.11
<200 mg/dL	8654 (55.47)	32,689 (56.50)	
200–239 mg/dL	5070 (32.50)	18,369 (31.75)	
≥240 mg/dL	1877 (12.03)	6796 (11.75)	
CCI score (*n*, %)			0.09
0	8533 (54.70)	36,099 (62.40)	
1	2649 (16.98)	8539 (14.76)	
≥2	4419 (28.33)	13,216 (22.84)	
Benign Prostate Hyperplasia (*n*, %)	3438 (23.40)	12,163 (20.70)	0.07

Abbreviations: CCI, Charlson comorbidity index; † obesity (BMI, body mass index, kg/m^2^) was categorized as <18.5 (underweight), ≥18.5 to <23 (normal), ≥23 to <25 (overweight), ≥25 to <30 (obese I), or ≥30 (obese II).

**Table 2:** Analyses of crude and overlap propensity score-weighted hazard ratios (95% confidence intervals) of gout for benign prostate hyperplasia.

	*N* of Event/ *N* of Total (%)	Follow-Up Duration (PY)	IR per 1000 (PY)	IRD (95% CI)	Hazard Ratios for Migraine			
					Crude †	*p* Value	Adjusted †,‡	*p*-Value
Total Participants								
Gout	3438/14,691 (23.40)	98,582	34.90	5.00 (3.72–6.16)	1.15 (1.11–1.20)	<0.001 *	1.13 (1.09–1.18)	<0.001 *
Control	12,163/58,764 (20.70)	406,328	29.90		1		1	
Age < 60 years old								
Gout	1862/7947 (23.43)	64,773	28.70	5.00 (3.68–6.37)	1.21 (1.15–1.27)	<0.001 *	1.19 (1.13–1.25)	<0.001 *
Control	6378/31,788 (20.06)	268,877	23.70		1		1	
Age ≥ 60 years old								
Gout	1575/6744 (23.35)	33,809	46.70	4.60 (2.03–6.96)	1.10 (1.04–1.16)	0.001 *	1.07 (1.01–1.13)	0.016 *
Control	5785/26,976 (21.44)	137,451	42.10		1		1	
Male								
Gout	3438/14,691 (23.40)	98,582	34.90	5.00 (3.72–6.16)	1.15 (1.11–1.20)	<0.001 *	1.13 (1.09–1.18)	<0.001 *
Control	12,163/58,764 (20.70)	406,328	29.90		1		1	
Low-income group								
Gout	1336/5953 (22.44)	38,036	35.10	6.40 (4.50–8.37)	1.22 (1.14–1.29)	<0.001 *	1.19 (1.12–1.27)	<0.001 *
Control	4538/23,812 (19.06)	158,159	28.70		1		1	
High-income group								
Gout	2102/8738 (24.06)	60,546	34.70	4.00 (2.42–5.57)	1.12 (1.07–1.12)	<0.001 *	1.10 (1.04–1.15)	<0.001 *
Control	7625/34,952 (21.82)	248,169	30.70		1		1	
Urban resident								
Gout	1546/6268 (24.66)	42,536	36.30	4.60 (2.73–6.56)	1.14 (1.07–1.20)	<0.001 *	1.12 (1.06–1.18)	<0.001 *
Control	5532/25,072 (22.06)	174,491	31.70		1		1	
Rural resident								
Gout	1892/8423 (22.46)	56,046	33.80	5.20 (3.57–6.74)	1.17 (1.11–1.23)	<0.001 *	1.15 (1.09–1.21)	<0.001 *
Control	6631/33,692 (19.68)	231,837	28.60		1		1	
Underweight								
Gout	33/173 (19.08)	913	36.10	7.00 (−4.72–18.78)	1.20 (0.83–1.72)	0.333	1.16 (0.81–1.68)	0.420
Control	259/1508 (17.18)	8896	29.10		1		1	
Normal weight								
Gout	746/3395 (21.97)	21,936	34.00	5.10 (2.71–7.60)	1.16 (1.07–1.25)	<0.001 *	1.13 (1.05–1.23)	0.002 *
Control	4014/20,146 (19.92)	139,116	28.90		1		1	
Overweight								
Gout	942/4067 (23.16)	27,398	34.40	3.70 (1.33–5.99)	1.11 (1.03–1.19)	0.005 *	1.08 (1.01–1.16)	0.035 *
Control	3584/16,689 (21.48)	116,657	30.70		1		1	
Obese								
Gout	1717/7056 (24.33)	48,335	35.50	5.10 (3.29–6.96)	1.16 (1.10–1.23)	<0.001 *	1.15 (1.09–1.22)	<0.001 *
Control	4306/20,421 (21.09)	141,659	30.40		1		1	
Nonsmoker								
Gout	1640/6226 (26.34)	41,741	39.30	5.80 (3.81–7.80)	1.29 (1.18 to 1.41)	<0.001 *	1.29 (1.20 to 1.38)	<0.001 *
Control	5592/24,436 (22.88)	167,011	33.50		1		1	
Past and current smoker								
Gout	1798/8465 (21.24)	56,841	31.60	4.10 (2.64–5.71)	1.17 (1.04 to 1.32)	0.011 *	1.19 (1.08 to 1.32)	<0.001 *
Control	6571/34,328 (19.14)	239,317	27.50		1		1	
Alcohol consumption < 1 time a week								
Gout	1642/6931 (23.69)	46,053	35.70	3.80 (1.93–5.56)	1.31 (1.20 to 1.43)	<0.001 *	1.26 (1.18 to 1.35)	<0.001 *
Control	6970/31,880 (21.86)	218,420	31.90		1		1	
Alcohol consumption ≥ 1 time a week								
Gout	1796/7760 (23.14)	52,529	34.20	6.60 (4.91–8.20)	1.22 (1.07 to 1.38)	0.002 *	1.23 (1.11 to 1.38)	<0.001 *
Control	5193/26,884 (19.32)	187,908	27.60		1		1	
SBP < 120 mmHg and DBP < 80 mmHg								
Gout	2102/9496 (22.14)	60,258	34.90	5.00 (3.40–6.48)	1.15 (1.10–1.21)	<0.001 *	1.05 (1.00–1.10)	0.050
Control	8497/42,344 (20.07)	283,778	29.90		1		1	
SBP ≥ 120 mmHg or DBP ≥ 80 mmHg								
Gout	1336/5195 (25.72)	38,324	34.90	5.00 (2.92–6.97)	1.16 (1.09–1.24)	<0.001 *	1.01 (0.94–1.07)	0.876
Control	3666/16,420 (22.33)	122,550	29.90		1		1	
Fasting blood glucose < 100 mg/dL								
Gout	1988/8084 (24.59)	57,414	34.60	4.40 (2.81–6.02)	1.14 (1.08–1.20)	<0.001 *	1.04 (0.99–1.09)	0.166
Control	7348/33,244 (22.10)	243,229	30.20		1		1	
Fasting blood glucose ≥ 100 mg/dL								
Gout	1450/6607 (21.95)	41,168	35.20	5.70 (3.81–7.59)	1.18 (1.12–1.25)	<0.001 *	1.02 (0.96–1.08)	0.567
Control	4815/25,520 (18.87)	163,099	29.50		1		1	
Total cholesterol < 200 mg/dL								
Gout	1779/7761 (22.92)	49,680	35.80	5.20 (3.51–6.96)	1.16 (1.10–1.22)	<0.001 *	1.01 (0.96–1.07)	0.663
Control	6875/33,582 (20.47)	224,898	30.60		1		1	
Total cholesterol ≥ 200 mg/dL								
Gout	1659/6930 (23.94)	48,902	33.90	4.80 (3.04–6.51)	1.16 (1.09–1.22)	<0.001 *	1.05 (0.99–1.11)	0.114
Control	5288/25,182 (21.00)	181,430	29.10		1		1	
CCI scores = 0								
Gout	1682/8225 (20.45)	56,651	29.70	3.50 (2.04–5.01)	1.14 (1.07–1.20)	<0.001 *	1.12 (1.06–1.18)	<0.001 *
Control	6851/36,407 (18.82)	261,857	26.20		1		1	
CCI scores = 1								
Gout	620/2410 (25.73)	16,241	38.20	4.50 (1.24–7.70)	1.17 (1.11–1.23)	<0.001 *	1.15 (1.09–1.21)	<0.001 *
Control	2029/8778 (23.11)	60,200	33.70		1		1	
CCI scores ≥ 2								
Gout	1136/4056 (28.01)	25,690	44.20	5.20 (2.46–8.06)	1.13 (1.06–1.21)	<0.001 *	0.98 (0.91–1.05)	0.485
Control	3283/13,579 (24.18)	84,271	39.00		1		1	

Abbreviations: IR, incidence rate; IRD, incidence rate difference; PY, person-year; * stratified Cox proportional hazard regression model, significance at *p* < 0.05. † Models were stratified by age, sex, income, and region of residence. ‡ The model was adjusted for age, sex, income, region, obesity status, smoking status, alcohol consumption, SBP, DBP, fasting blood glucose, total cholesterol, and CCI score.

## Data Availability

Restrictions apply to the availability of these data. Data was obtained from the Korean National Health Insurance Service-Health Screening Cohort and are available from https://nhiss.nhis.or.kr/bd/ab/bdaba021eng.do, accessed on 22 December 2023, with the permission of Korean National Health Insurance Service.
